# Characteristics and Outcomes of Shared Bicycle-Related Injuries from a Large Emergency Medical Centre in China, 2017–2021

**DOI:** 10.1155/2022/4647102

**Published:** 2022-06-22

**Authors:** Mao Chen, Weiwei Li, Jun Ye, Gang Liu, Chaolin Huang

**Affiliations:** ^1^Department of Emergency Medicine, The First Affiliated Hospital of Chengdu Medical College, Chengdu, China; ^2^Department of General Surgery, The First People's Hospital of Chengdu City, Chengdu, China; ^3^Department of Clinical Laboratory, The Second Affiliated Hospital of Guizhou Medical University, Kaili, China; ^4^Department of Medical Administration, The First Affiliated Hospital of Chengdu Medical College, Chengdu, China; ^5^Department of Gynaecology, The First Affiliated Hospital of Chengdu Medical College, Chengdu, China

## Abstract

**Objective:**

The aim of this study is to investigate the characteristics and outcomes of shared bicycle-related injuries from a large emergency medical centre in China in five years from January 2017 to December 2021.

**Methods:**

This study was conducted by reviewing the electronic medical record database of a large hospital in China for cases of shared bicycle-related injuries in five years from January 2017 to December 2021. The collected information included demographic data, injury characteristics, and outcomes. Multivariate logistic regression analysis was used to identify risk factors for fatal injury among victims.

**Results:**

Most shared bicycle-related injuries occurred in male (60.50%), aged 18–35 (38.81%). Company employees (29.28%) were the majority of victims of shared bicycle-related injuries. Riding in a motor vehicle lane was the most common unsafe riding behaviour (26.52%). The lower limb was the most frequently injured body region (25.28%). Bruising (28.73%) was the most commonly diagnosed injury type. The fatality rate was 9.53%, 72.24% of victims recovered well without permanent disability, and 18.23% of victims had permanent disabilities. The length of hospital stay of most of the victims (67.54%) was less than 7 days, and the hospitalization cost of most of the victims (51.93%) was less than 20,000 Yuan. Riding in a motor vehicle lane, running red lights, and cycling against traffic flow are risk factors for fatal injury.

**Conclusions:**

This study indicated that shared bicycle-related injuries make up a sizeable proportion of injuries presenting to the emergency department and with diverse injury characteristics and outcomes. The findings reflect that shared bicycle-related injury has become a public health problem. Therefore, it is necessary to establish injury prevention strategies for the safety of shared bicycle users.

## 1. Introduction

As a convenient, low-cost, and environmentally friendly mode of transport, shared bicycles have developed rapidly in China in recent years [1, 2]. Shared bicycles work as short-term bicycle rental services based on GPS and smartphone technology. It is convenient to use, and it requires only a smartphone to unlock a shared bicycle and pay the fees [3, 4]. By March 2020, 16 million shared bicycles had been launched in Chinese cities, and users could rent and return shared bicycles almost anywhere [5]. According to the China Academy of Information and Communications Technology, there were 221 million registered shared bicycle users by the end of 2017 [6]. Shared bicycles effectively fill the so-called last-mile traffic gap between work and home locations and metro stations for city commuters. In China's large cities with heavy traffic congestions and under environmental stress due to air pollution, shared bicycle services combined with well-developed metro systems provide a convenient, efficient, low-cost, and environmentally friendly travel solution [7–9].

In China, approximately 8.5% of road traffic deaths and 19.1% of road injuries occurred among cyclists in 2017 [8]. However, shared bicycle use presents somewhat different risks compared with private bicycles, as their use may be for short-distance efficient commuting in large cities with heavy traffic rather than long-distance riding for pleasure or exercise in countryside. There are few studies that focused on shared bicycle-related injuries in China. One study was conducted by WeChat software-based online survey and found that shared bicycle-related injuries are associated with unsafe riding behaviours including running red light, cycling against the traffic flow, carrying passengers, and distracted riding [8]. However, the study did not include the patterns of injuries and clinical outcomes of the victims, which are also essential parts of shared bicycle-related injuries. Another study conducted in 2017, when shared bicycles just began to be implemented in China, may not represent the real situation of shared bicycle use at present [10].

For planning and implementing effective interventions to prevent shared bicycle-related injuries, it is essential to fully understand how shared bicycle-related injuries occur and their severities and types. In this study, we aimed to explore the prevalence, injury patterns, and outcomes of shared bicycle-related injuries presenting to the emergency department of a large hospital in China. Analysis and study of the characteristics and outcomes of shared bicycle-related injuries will be helpful in providing support for the prevention and treatment of shared bicycle-related injuries.

## 2. Materials and Methods

### 2.1. Study Design and Participants

Chengdu is the capital city of Sichuan Province and the largest city in southwestern China, with a population of 20.93 million spread over an area of 14,335 km^2^. The First People's Hospital of Chengdu city is the largest tertiary hospital in Chengdu, with 3000 inpatient beds, and more than 1800,000 patients visit the hospital every year. The hospital is also the emergency medical centre of Chengdu city, and it undertakes emergency services for 20.93 million people living in the city and its surrounding suburbs. This study was conducted by reviewing the electronic medical record database of The First People's Hospital of Chengdu city in five years from January 2017 to December 2021.312,351 patients visited the emergency department during the study period. 16,117 cases were identified according to ICD-10 codes relating to trauma or injury. The inclusion criteria were trauma or injury involved with shared bicycle and complete the treatment in this hospital. The exclusion criteria were incomplete information, and drunk driving of the wrecker or drunk riding of the shared bicycle users. At last, 724 cases involved with shared bicycle injuries were included in the present study. The flowchart of the study is shown in Figure 1. Ethics approval for this study was obtained from the Ethics Committee of The First People's Hospital of Chengdu city.

### 2.2. Data Collection

Demographic data, including age, gender, education level, and occupation, were extracted from the electronic medical record database. Incident-related data included the time and condition of the victim, while the occurrence of injuries and injury-related data, including the type of injury, the region of injury, severity of the injury, clinical outcomes, length of hospital stay, and hospitalization cost, were also extracted from the electronic medical record database. The severity of the injury was determined using the Kampala Trauma Score II (KTS II) [11].

### 2.3. Statistical Analysis

Data entry was performed using Excel 2010 (Microsoft Corp., Redmond, WA), and data analysis was conducted using IBM SPSS version 20.0 (IBM, Armonk, NY). Multivariate logistic regression modelling was used to calculate adjusted odds ratios (ORs) with 95% confidence intervals (CIs) to identify risk factors for fatal injury. A *P* value <0.05 was considered statistically significant.

## 3. Results

### 3.1. The Overall Trend and Demographical Characteristics of Shared Bicycle-Related Injuries

A total of 312,351 patients visited the emergency department from January 2017 to December 2021. There were 16,117 cases related to trauma or injury, of which 724 (4.49%) cases involved with shared bicycle injuries were included in the present study. The flowchart of the study is shown in Figure 1. The trend of shared bicycle-related injuries was increased during the study period from 105 in 2017 to 184 in 2021 (Figure 2).  Table 1 provides the demographical characteristics of these cases. Among the 724 patients treated for shared bicycle-related injuries, male had a higher proportion (60.50%) than female (39.50%). The highest proportion of victims was young adults aged 18–35 (38.81%), followed by adults aged 36–45 (28.87%). Regarding educational status, victims with higher education ranked first (37.71%), followed by high school (28.04%) and middle school (19.61%). The majority of the victims were company employees (29.28%) followed by daily labourers (21.27%) (Table 1).

### 3.2. Time and Situations of the Victims during the Occurrence of Shared Bicycle-Related Injuries

The majority of shared bicycle-related injuries occurred in the morning (7 : 00–9:00) (33.57%) and in the evening (17 : 00–19 : 00) (31.08%), coinciding with the morning and afternoon rush hour. Regarding the situations of the victims during the occurrence of shared bicycle-related injuries, the most common was riding in a motor vehicle lane (26.52%), followed by running red lights (21.27%), using a cell phone while riding (13.54%), cycling against the traffic flow (11.46%), eating while riding (10.50%), and carrying passengers (10.36%). The most common mechanism of injury were collisions with motor vehicles (56.91%), while 28.18% were single bicycle crashes. Collisions with other bicycles and pedestrians were rare (Table 2).

### 3.3. Characteristics of Shared Bicycle-Related Injuries

Bruising (28.73%) was the most commonly diagnosed injury type, followed by contusion (26.52%) and fracture (17.54%). Less common injury types were dislocation (13.12%) and open wounds (10.77%). The lower limb was the most frequently injured body region (25.28%), followed by the head (22.37%) and upper limb (16.30%). Multiple regions injury (10.22%), neck injury (10.91%), and trunk injury (14.92%) were less frequently occurred. According to the Kampala Trauma Score II (KTS II) classification of trauma severity, mild injuries (KTS II = 9–10) accounted for 48.62%, moderate injuries (KTS II = 7–8) accounted for 29.56% and severe injuries (KTS II ≤ 6) accounted for 21.82% (Table 3).

### 3.4. Clinical Outcomes and Hospitalization Characteristics of Shared Bicycle-Related Injuries

Out of the 724 victims studied, the fatality rate was 9.53% and the cause of the fatality was that the shared bicycle riders were run down by motor vehicles. Among the victims who survived, 72.24% recovered well without permanent disability, but 18.23% were left with permanent disabilities because of amputation or severe spinal cord injury. The length of hospital stay of most of the victims (67.54%) was less than 7 days, and the hospitalization cost of most of the victims (51.93%) was less than 20,000 Yuan. However, the length of hospital stay of 10.77% victims was more than 14 days, and the hospitalization cost of 12.02% victims was more than 50,000 Yuan (Table 4).

### 3.5. Multivariate Logistic Regression Analysis to Identify Risk Factors for Fatal Injury among Victims

Multivariate regression analysis was performed to identify risk factors for fatal injury. According to the multivariate regression analysis, a 10.25-fold (95%CI: 7.91 to 15.23; *p* = 0.005) higher risk of fatal injury was found for shared bicycle users riding in a motor vehicle lane relative to normal riding. Also, the results show that running red lights and cycling against traffic flow increased the risk of fatal injury. About 12.01-fold (95% CI: 6.83–17.01; *p* = 0.017) and 7.53-fold (95% CI: 2.81–11.27; *p* = 0.014) higher risks of fatal injury were seen for shared bicycle users running red lights and cycling against traffic flow relative to normal riding, respectively (Table 5). No differences in the risk of fatal injury were observed based on gender, age, educational status, occupation, and occurrence time.

## 4. Discussion

This study focused on the characteristics and outcomes of shared bicycle-related injuries from a large emergency medical centre in China. Findings from this study may provide useful data for planning and implementing effective interventions to prevent shared bicycle-related injuries.

The present study showed that the majority of victims were young people, and most of them were male. Our results are consistent with previous studies showing that gender and age are among the main factors associated with bicycle-related injuries [12–14]. We also found that company employees and people with higher education are the majority of victims of shared bicycle-related injury. In China, people with higher education usually work as company employees in large cities. In regard to heavy traffic congestions and well-developed metro systems in large Chinese cities, taking metro systems is more convenient than driving a car in rush hours [15, 16]. Company employees effectively use shared bicycles to fill the so-called last-mile traffic gap between work and home locations and metro stations [17–19].

Our findings suggested that the peak time of shared bicycle-related injury occurred during the rush hours for the working force, similar to the injuries previously reported in other studies [10, 20]. This result implies that shared bicycle users should use protective measures such as reflective clothing and helmets while riding in heavy traffic flows during rush hours [21]. This study also revealed that most of the shared bicycle-related injuries were caused by unsafe riding behaviours [8, 22]. These unsafe riding behaviours include riding in a motor vehicle lane, using a cell phone while riding, cycling against the traffic flow, eating while riding, running red lights, and carrying passengers. We conjectured that this might be due to a sense of “time urgency” in shared bicycle users. Because most shared bicycle users are city commuters, they hastily ride shared bicycles between work and home locations and subway stations. More than half of all hospitalized injuries occurred due to collision with motor vehicles, while 28.18% of injuries were single bicycle crashes. These findings suggest that safety education should be carried out among shared bicycle users and motor vehicle drivers.

The head and extremities were the most common body regions injured in the present study, both of which were significantly associated with injury severity and death [18, 23]. Therefore, protective measures such as helmets, knee pads, and elbow pads should be mandatory for shared bicycle users. Most of the victims suffered from mild injuries with good clinical outcomes. However, 9.53% of victims were dead and 18.23% of victims were left with permanent disabilities. It is very important that doctors take adequate treatment measures to prevent injury deteriorate and death occurs while victims present to emergency centres. Additionally, passive preventive strategies should be taken to lower the rates of shared bicycle-related injury. For example, wheels with spoke covers could prevent extremities from getting caught in the spokes and energy-absorbing handlebars could avoid abdominal injuries [24]. Speed limit could reduce impact force and severity of injury.

According to our multivariate analysis for predicting fatal injury, riding in a motor vehicle lane, running red lights, and cycling against traffic flow are risk factors for fatal injury. These unsafe riding behaviours increase the risk of being hit by motor vehicles, thus sustaining a fatal injury [25]. Therefore, it is very important to raise safety awareness when using shared bicycles.

This study has some limitations. The study cases were identified by reviewing the electronic medical record database of a single-centre; it is possible that some bicycle-related injury cases were not included. There were patients treated in other healthcare settings, and those who did not receive medical attention were not included in the electronic medical record database. Consequently, our data might underestimate the prevalence and magnitude of the problem. Despite its limitations, we believe our results could contribute to better understanding of the characteristics and outcomes of shared bicycle-related injuries in China, which may provide useful and valuable information to develop injury prevention measures.

## 5. Conclusions

This study indicated that shared bicycle-related injuries make up a sizeable proportion of injuries presenting to the emergency department and with diverse injury characteristics and outcomes. The findings reflect that shared bicycle-related injury has become a public health problem. Therefore, it is necessary to establish injury prevention strategies for the safety of shared bicycle users. The implementation of policies such as compulsory helmet use and safety education among shared bicycle users should be considered to improve the current situation of shared bicycle-related injuries in China.

## Figures and Tables

**Figure 1:** Flowchart of the study.

**Figure 2:** The trend of shared bicycle-related injuries increased during the study period from 105 in 2017 to 184 in 2021.

**Table 1:** Demographical characteristics of patients with shared bicycle-related injuries.

Variables	Frequency (*N* = 724)	Percentage (%)
Gender		
Male	438	60.50
Female	286	39.50

Age		
14–17	98	13.54
18–35	281	38.81
36–45	209	28.87
≥46	136	18.78

Educational status		
Primary school	106	14.64
Middle school	142	19.61
High school	203	28.04
Higher education	273	37.71

Occupation		
Student	103	14.23
Teacher	87	12.02
Doctor	46	6.35
Businessman	83	11.46
Daily labourer	154	21.27
Company employee	212	29.28
Others	39	5.39

**Table 2:** Time and conditions of the victims during the occurrence of shared bicycle-related injuries.

Variables	Frequency (*N* = 724)	Percentage (%)
Occurrence time		
7 : 00–9:00	243	33.57
10 : 00–12 : 00	131	18.09
13 : 00–15 : 00	78	10.77
17 : 00–19 : 00	225	31.08
Others	47	6.49

Condition of the victim		
Normal riding	14	1.93
Riding in a motor vehicle lane	192	26.52
Running red lights	154	21.27
Using a cell phone	98	13.54
Cycling against traffic flow	83	11.46
Eating while riding	76	10.50
Carrying passengers	75	10.36
Others	32	4.42

Mechanism of injury		
Collision with motor vehicle	412	56.91
Single bicycle crash	204	28.18
Collision with another bicycle	58	8.01
Collision with pedestrian	35	4.83
Others	15	2.07

**Table 3:** Characteristics of shared bicycle-related injuries.

Variables	Frequency (*N* = 724)	Percentage (%)
Injury type		
Fracture	127	17.54
Bruise	208	28.73
Contusion	192	26.52
Dislocation	95	13.12
Open wound	78	10.77
Others	24	3.32

Injured body region		
Head	162	22.37
Neck	79	10.91
Trunk	108	14.92
Upper limb	118	16.30
Lower limb	183	25.28
Multiple region	74	10.22

Kampala Trauma Score II		
9-10	352	48.62
7-8	214	29.56
≤6	158	21.82

**Table 4:** Clinical outcomes and hospitalization characteristics of shared bicycle-related injuries.

Variables	Frequency (*N* = 724)	Percentage (%)
Clinical outcomes		
Fatality	69	9.53
Left with permanent disabilities	132	18.23
Recovered without permanent disability	523	72.24

Length of hospital stay (days)		
≤7	489	67.54
8–14	157	21.69
≥14	78	10.77

Hospitalization cost (Yuan)		
≤20,000	376	51.93
20,000–50,000	261	36.05
≥50,000	87	12.02

**Table 5:** Results of multivariate logistic regression analysis on fatal injury versus nonfatal injury.

Risk factor	Unadjusted		Adjusted	
	OR (95% CI)	*P* value	OR (95% CI)	*P* value
Gender				
Female	1.00 (reference)		1.00 (reference)	
Male	1.53 (0.63, 3.48)	0.101	0.93 (0.43, 4.23)	0.241

Age				
14–17	1.00 (reference)		1.00 (reference)	
18–35	1.92 (0.68, 4.83)	0.117	0.95 (0.71, 4.02)	0.213
36–45	1.01 (0.76, 3.89)	0.123	1.43 (0.82, 3.14)	0.141
≥46	0.76 (0.24, 2.53)	0.132	0.82 (0.36, 2.69)	0.232

Educational status				
Primary school	1.00 (reference)		1.00 (reference)	
Middle school	0.73 (0.33, 4.76)	0.142	0.85(0.47, 5.81)	0.274
High school	1.93 (0.34, 6.91)	0.173	1.07(0.15, 6.92)	0.265
Higher education	0.82 (0.27, 5.96)	0.241	0.90(0.31, 7.32)	0.371

Occupation				
Student	1.00 (reference)		1.00 (reference)	
Teacher	0.64 (0.16, 5.32)	0.165	0.77(0.27, 6.32)	0.357
Doctor	1.75 (0.14, 7.28)	0.261	1.04(0.46, 5.26)	0.217
Businessman	0.65 (0.13, 4.37)	0.115	1.13(0.37, 6.82)	0.152
Daily labourer	1.82 (0.17, 6.32)	0.127	0.65(0.43, 4.31)	0.315
Company employee	0.73 (0.46, 7.27)	0.232	0.72(0.14, 9.86)	0.452
Others	0.33 (0.19, 5.48)	0.171	0.87(0.17, 7.85)	0.552

Condition of the victim				
Normal riding	1.00 (reference)		1.00 (reference)	
Riding in a motor vehicle lane	11.14 (7.31, 17.26)	0.001	10.25 (7.91, 15.23)	0.005
Running red lights	13.2 (5.94, 20.16)	0.012	12.01 (6.83, 17.01)	0.017
Using a cell phone	1.13 (1.84, 8.21)	0.102	1.28 (2.34, 7.87)	0.125
Cycling against traffic flow	8.34 (1.31, 13.32)	0.021	7.53 (2.81, 11.27)	0.014
Eating while riding	1.12 (1.07, 10.21)	0.214	2.39 (1.85, 8.79)	0.326
Carrying passengers	1.78 (0.95, 9.27)	0.132	1.08 (1.97, 8.07)	0.147
Others	1.37 (1.94, 7.24)	0.208	1.06 (0.91, 5.21)	0.326

Occurrence time				
7 : 00–9:00	1.00 (reference)		1.00 (reference)	
10 : 00–12 : 00	0.37 (0.12, 3.15)	0.112	0.41 (1.19, 3.11)	0.217
13 : 00–16 : 00	1.15 (0.09, 2.78)	0.332	1.22 (0.12, 2.14)	0.323
17 : 00–19 : 00	2.83 (0.16, 2.63)	0.405	2.87 (0.19, 2.27)	0.417
Others	0.07 (0.03, 2.14)	0.171	0.09 (0.04, 2.01)	0.223

## Data Availability

The data used to support the findings of this study are available from the corresponding author upon request.
